The article "Sales Forecast of Marketing Brand Based on BP Neural Network Model" was retracted in 2023. Reasons: signs of a paper mill; suspected computer-generated content; unreliable results or conclusions; concerns about the data.

# Sales Forecast of Marketing Brand Based on BP Neural Network Model

**DOI:** 10.1155/2022/1769424

**Published:** 2022-06-28

**Authors:** Wei Feng

**Affiliations:** College of International Education, Jiangsu Vocational College of Finance and Economics, Huaian 223003, Jiangsu, China

## Abstract

With the advancement of globalization, the market competition among enterprises has become increasingly intense. To win a good market, an enterprise must understand and grasp the laws of the market economy and accordingly predict the future of the market. Efficient market estimates are based on a careful study of various types of market data. Therefore, enterprises must engage in preliminary research and data collection, based on a complete data system, and ensure the accuracy of vision predictions by developing a scientific market vision. Only by ensuring correct estimates can companies develop a right business plan and ultimately capture the market. More traditional sales forecasting methods generally only involve some details of sales, not accounting for relatively complex interactions among those factors (price, consumer income, etc.) that affect demand, and as a result, the models built are relatively simple. Artificial neural networks have excellent capabilities for infinite mapping and passive learning. This affects the requirements among the various factors, as well as the more complex relationships between them. In terms of weights, it is safe for neural networks. Therefore, BP neural network technology is used by most people to predict the number of sales, and a more coherent sales forecast method has been established for this purpose. Predicting sales targets is a very complex process, as the experimental results show. The prediction accuracy of this model is much higher than that of other common prediction methods. Its prediction accuracy is more than 30% higher than that of conventional methods, and it also has better comprehensive performance. This has a certain application value for sales forecasting work.

## 1. Introduction

In recent years, the contradiction between production and sales has become increasingly prominent. Sometimes the brand sells well, and the production and sales of branded goods may not be balanced, resulting in insufficient supply. Or affected by market failure, the sales of branded products will decline, resulting in excess production capacity and a large waste of resources. In addition, due to market fluctuations, the sales of branded products must be precisely controlled, and the production quantity will be difficult to grasp, so this will bring certain economic losses to the enterprise. Therefore, to minimize this economic loss, it is necessary to forecast the sales of the brand, while the enterprise develops a reasonable amount of goods production.

The article "Sales Forecast of Marketing Brand Based on BP Neural Network Model" was retracted in 2023. Reasons: signs of a paper mill; suspected computer-generated content; unreliable results or conclusions; concerns about the data.

The research significance of this paper is to provide a certain scientific basis for enterprises in the decision-making of sales quantity management and their daily production and operation activities. Today, it is increasingly difficult for companies to survive. Therefore, the marketing strategy formulated by an enterprise must be based on real and reliable data and accurately predict the development trend of the future market, to improve the accuracy of the most important decision-making processes in an enterprise. In addition, enterprises often need to optimize the internal structure in the process of development. The research content of this paper can also provide some technical support for enterprises to improve the work efficiency. It can also effectively prevent and mitigate many bad influences, to realize the company's vision of stable and rapid development in the future market.

This paper selects the sales data of a factory for analysis and then uses the neural network forecasting method and the linear mapping method to forecast the sales quantity, to analyze the accuracy and reliability of the two methods. For neural network and sales forecasts, there is no preference of one over the other, and a detailed analysis of each is carried out to make the content of the article more complete.

## 2. Related Work

For BP neural network, domestic and foreign experts have conducted extensive researches. Based on experimental data, Ma et al. established a BP neural network prediction model for determining the heat transfer coefficient of supercritical water. The results show that the trained BP neural network prediction model can better predict and understand the heat transfer coefficient of supercritical water [1]. Li et al. proposed a new method that combines chaotic algorithm with genetic algorithm (CGA). The basic idea is to encode the weights and thresholds of the BP neural network and use the genetic algorithm to obtain a general optimal solution. Simulation and experimental results show that the real-time performance and accuracy of gesture recognition have been greatly improved after using CGA [2]. Wang et al. adopted MEA's BP Neural Network (BPNN) to improve the generalization ability and predictability of BPNN. Research results show that MEA-BP outperforms GA-BP and standard BP neural network model (St-BP) with faster running time and higher prediction accuracy [3]. For sales forecasting, Hung et al. developed a sales forecasting model that analyzes the interaction of two forms of retail competition (convenience-oriented and budget-oriented). The traditional method for making such predictions is based on the Lotka–Volterra equation (also known as the LV model) [4]. Stormi et al. studied installed-base information to help service original equipment manufacturers (OEMs) predict and support their industrial service sales, thereby improving OEMs' understanding of their customer lifetime value (CLV) dynamics [5].

The article "Sales Forecast of Marketing Brand Based on BP Neural Network Model" was retracted in 2023. Reasons: signs of a paper mill; suspected computer-generated content; unreliable results or conclusions; concerns about the data.

## 3. Neural Network Model

The sales volume of a product is closely related to and inseparable from its market demand. The changes in the demand and quantity of the market are also very complex and elusive. The factors (price, demand, etc.) that can affect the volume of sales of a company's products are numerous and difficult to control. At least against the economic background of the current technical level, it is difficult to establish a relatively accurate mathematical model to predict the sales volume of enterprise products. However, it is possible to make predictions in the range direction, and it is not impossible to predict values close to the true value [6–8]. Therefore, many people are now focusing on the field of neural networks, because this field has very obvious and incomparable advantages in solving some difficult and numerically missing problems.

### 3.1. Theoretical Basis of BP Network Model

The BP neural network model is composed of several parallel and distributed numerical processors composed of some relatively simple processing numerical units. Numerical processors of this type have the natural characteristics of storing values and have empirical knowledge in the application inventory. The network is similar to the human brain; this similarity can be roughly summarized in two aspects. On the one hand, the neural network is used in the learning process to acquire some knowledge related to the external environment. On the other hand, internal neurons can be used to store information about the knowledge gained in relation to numerical processing [9]. The most commonly used neural network model is the M-P model. Its details are shown in Figure 1.

The main purpose of artificial neurons is to construct a neuron network [10]. And when building a neuron network, the main consideration for choosing which neuron to build is to see what effect the neuron function can simulate. Its characteristics are as follows: 1. distributed storage of information; 2. strong adaptability; 3. capability of parallel processing; 4. content addressable memory function; 5. automatic extraction of characteristic parameters; 6. fault tolerance [11].

The research content and direction of neural network are quite large. The research content concerns almost all walks of life, such as industry, commerce, and animal husbandry, which perfectly reflects the characteristics of interdisciplinary and cross-industry integration of other technical fields [12]. Due to space problems, the typical 13 network models cannot be counted. Only a few of the more commonly used neural network models are introduced here.

1. BP neural network is also called “error backpropagation training artificial neural network.” It uses the error between the output response of the network to the learning signal and the expectation as a mentor signal to adjust the network connection strength. It is adjusted repeatedly to minimize the error, thus completing the learning process. The schematic diagram of its specific process structure is shown in Figure 2.
2. Hopfield neural network is a kind of neural network that can feed back information, being a kind of partial dynamic neural network. It not only has to input and output data at the same time, but also has to wait for a period of time to have a relatively stable effect [13]. The network can be divided into two types: discrete networks and continuous networks. Among them, discrete networks can be used in associative memory, while continuous networks are mainly used in optimization calculations. The specific schematic diagram is shown in Figure 3.

The article "Sales Forecast of Marketing Brand Based on BP Neural Network Model" was retracted in 2023. Reasons: signs of a paper mill; suspected computer-generated content; unreliable results or conclusions; concerns about the data.

### 3.2. Algorithm of BP Network Model

Thus far, the multilayer network model using the BP algorithm is the most widely used neural network model, it includes three-layer network model and seven-layer network model, and a single hidden layer network is the most widely used among such networks [14].

The following is a simple analysis of the mathematical relationship between the signals of each layer.

For the output layer, *A* is the output value, and there are

(1) $$\begin{array}{c} A_{i}=f\left({\text{net}}_{i}\right),i=1,2,\ldots ,i,\\ {\text{net}}_{i}=\sum_{j=0}^{m}u_{ji}y_{j},\;i=1,2,\ldots ,i. \end{array}$$

For the hidden layer, there are

(2) $$\begin{array}{c} y_{j}=f\left({\text{net}}_{j}\right),\;j=1,2,\ldots ,m,\\ {\text{net}}_{j}=\sum_{i=0}^{n}v_{ij}x_{i},\;j=1,2,\ldots ,m. \end{array}$$

Then, the unipolar function is

(3) $$\begin{array}{c} f\left(x\right)=\frac{1}{1+e^{-x}}, \end{array}$$

and *f*(*x*) has the characteristics of continuous and derivation; then,

(4) $$\begin{array}{c} f{\;}^{\prime }\left(x\right)=f\left(x\right)\left[1-f\left(x\right)\right]. \end{array}$$

The bipolar function is

(5) $$\begin{array}{c} f\left(x\right)=\frac{1-e^{-x}}{1+e^{-x}}. \end{array}$$

When the actual output value is not equal to the expected output value, there is an output error *W*, which is

(6) $$\begin{array}{c} W=\frac{1}{2}{\left(d-o\right)}^{2}=\frac{1}{2}\sum_{i=1}^{i}{\left(d_{i}-o_{i}\right)}^{2}. \end{array}$$

The formula expanded to the hidden layer is

(7) $$\begin{array}{c} W=\frac{1}{2}\sum_{i=1}^{i}{\left[d_{i}-f\left({\text{net}}_{i}\right)\right]}^{2}=\frac{1}{2}\sum_{i=1}^{i}{\left[d_{i}-f\left(\sum_{j=0}^{m}u_{ji}y_{j}\right)\right]}^{2}. \end{array}$$

It expands to the input layer as

(8) $$\begin{array}{c} W=\frac{1}{2}\sum_{i=1}^{i}{\left\{d_{i}-f\left[\sum_{j=0}^{m}u_{ji}f\left({\text{net}}_{j}\right)\right]\right\}}^{2}=\frac{1}{2}\sum_{i=1}^{i}{\left\{d_{i}-f\left[\sum_{j=0}^{m}u_{ji}f\left(\sum_{l=0}^{n}v_{lj}x_{l}\right)\right]\right\}}^{2}. \end{array}$$

The adjustment amount and the negative gradient of the error are

(9) $$\begin{array}{c} \Delta u_{ji}=-\eta \frac{\partial W}{\partial u_{ji}},\;j=0,1,2,\ldots ,m;\;i=1,2,\ldots ,i,\\ \Delta v_{ij}=-\mu \frac{\partial W}{\partial v_{lj}},\;l=0,1,2,\ldots ,n;\;j=1,2,\ldots ,m. \end{array}$$

The adjustment formula is

(10) $$\begin{array}{c} \phi_{i}^{o}=\left(d_{i}-o_{i}\right)o_{i}\left(1-o_{i}\right),\\ \phi_{j}^{y}=\left[\sum_{i=1}^{i}\left(d_{i}-o_{i}\right)f\prime \left({\text{net}}_{i}\right)u_{ji}\right]f\prime \left({\text{net}}_{j}\right)=\left(\sum_{i=1}^{i}\phi_{i}^{o}u_{ji}\right)y_{j}\left(1-y_{j}\right),\\ \Delta u_{ji}=\eta \phi_{i}^{o}y_{j}=\eta \left(d_{i}-o_{i}\right)o_{i}\left(1-o_{i}\right)y_{j},\\ \Delta V_{lj}=\eta \phi_{j}^{y}x_{l}=\eta \left(\sum_{i=1}^{i}\phi_{i}^{o}u_{ji}\right)y_{j}\left(1-y_{j}\right)x_{l}. \end{array}$$

The weight formula of the output layer is

(11) $$\begin{array}{c} \Delta u_{ji}^{h+1}=\eta \phi_{i}^{h+1}y_{j}^{h}=\eta \left(d_{i}-o_{i}\right)o_{i}\left(1-o_{i}\right)y_{j}^{i},\;j=0,1,2,\ldots ,m_{h};\;i=1,2,\ldots ,i. \end{array}$$

The weight formula of the hidden layer is

(12) $$\begin{array}{c} \Delta u_{lj}^{h}=\eta \phi_{j}^{h}y_{l}^{h-1}=\eta \left(\sum_{i=1}^{i}\phi_{i}^{o}u_{ji}^{h+1}\right)y_{j}^{h}\left(1-y_{j}^{h}\right)y_{l}^{h-1},\;i=0,1,2,\ldots ,m_{h-1};\;j=1,2,\ldots ,m_{h}. \end{array}$$

The vector form of the output layer is

(13) $$\begin{array}{c} Y={\left(y_{0},y_{1},y_{2},\ldots ,y_{j},\ldots ,y_{m}\right)}^{T},\\ \phi^{o}={\left(\phi_{1}^{o},\phi_{2}^{o},\ldots ,\phi_{i}^{o},\ldots ,\phi_{l}^{o}\right)}^{T}. \end{array}$$

Then,

(14) $$\begin{array}{c} \Delta U=\eta {\left(\phi^{o}Y^{T}\right)}^{T}. \end{array}$$

The vector form of the hidden layer is

(15) $$\begin{array}{c} X={\left(x_{0},x_{1},x_{2},\ldots ,x_{i},\ldots ,x_{n}\right)}^{T},\\ \phi^{y}={\left(\phi_{1}^{y},\phi_{2}^{y},\ldots ,\phi_{j}^{y},\ldots ,\phi_{m}^{y}\right)}^{T}. \end{array}$$

Then,

(16) $$\begin{array}{c} \Delta V=\eta {\left(\phi^{y}X^{T}\right)}^{T}. \end{array}$$

The article "Sales Forecast of Marketing Brand Based on BP Neural Network Model" was retracted in 2023. Reasons: signs of a paper mill; suspected computer-generated content; unreliable results or conclusions; concerns about the data.

### 3.3. Process of BP Network Model

The characteristics of the BP algorithm are the forward calculation of the signal and the backpropagation of the error [15]. The specific flow of the algorithm signal is shown in Figure 4.

### 3.4. EBP Neural Network

EBP neural network is also known as backpropagation network [16]. The introduction of hidden layer neurons improved the classification and memory capabilities of neural networks, and researchers began to focus on hidden layer neurons. The EBP algorithm (BP for short) was written in this context. In addition, the BP network also overcomes technical problems that XOR and other simple perceptrons cannot solve. Therefore, the BP model is recognized and accepted by most researchers, and it has also become one of the typical models of neural network models. Since then, it has played an important role in neural networks.

The neural network is further divided into single-layer and multilayer network, and the specific structure diagram is shown in Figure 5.

In practical applications, the most widely used is the multilayer neuron network. The following takes the schematic diagram of the three-layer neuron network model structure as an example, as shown in Figure 6.

This network model is different from other models. The state of the neurons in this layer of the model will only affect the state of the neurons in the present layer and will not continue to affect the state of the neurons in the next layer. In other words, the state of the neuron is only affected by the hierarchy, and the effect does not go beyond the layer. In the model structure, after the signal is transmitted to the output layer, when the desired output result is not received, the output signal will start to back propagate. That is, it goes back along the original output channel and delivers an error-generating signal. The weight of each neuron changes layer by layer to minimize the value of the mean square value of the final output error. Since neurons restrict and affect each other, there is a high degree of nonlinearity between the input and output, so neurons can be used for function approximation and curve fitting [17, 18].

## 4. Sales Forecast Experiment

When making sales forecasts for the present, qualitative decisions can be made based on experience. The forecast for current sales can also use mathematical methods to quantitatively process historical data and establish prediction models for scientific prediction. Empirical forecasting methods are often used to forecast small amounts of data. Because their advantage is to draw on experience when making judgments, decisions can be made faster and results can be obtained quickly. However, the prediction results are often subjective, and quantitative models are divided into time series models, causal models, and mixed models.

The article "Sales Forecast of Marketing Brand Based on BP Neural Network Model" was retracted in 2023. Reasons: signs of a paper mill; suspected computer-generated content; unreliable results or conclusions; concerns about the data.

A good sales forecast is essential to improve the company's profitability and economic efficiency [19]. According to the constructed model, the specific steps of using BP neural network to predict the time series of the sales volume of the switch factory are as follows:

1. It selects the required sample data and builds a sample analysis model. As of 2020, the annual switch sales of switch factories were performed in the past 20 years. At the same time, the annual price index and income index are obtained according to the China Statistical Yearbook. The results are shown in Table 1.
2. Data is classified into sample data and test data. Firstly, the collected data is simply classified, and the sales data of switch factories from 2001 to 2016 is used as sample data. The data of the next few years is used as the test data for the prediction ability of the neural network, and the data is classified into sample data and test data.
3. The sample data is preprocessed: the data in the table is normalized according to the previous model and formula.
4. The number of network layers and the number of hidden layer neurons are preliminarily determined. Neural networks can show the relationship between the number of sales, the sales price, and the sales revenue. The network model has a total of 2 input nodes, 6 hidden layer nodes, and 1 output node. The two input nodes represent the sales price and sales revenue, and the output node represents the sales quantity.

Based on the data from 2001 to 2016 as the modeling basis, the data from 2017 to 2020 can be forecast. After many trials, the root mean square error (input normalized sample) can reach 0.0002. At this point, the network model representation can also estimate all sample points. In other words, the neural network has successfully realized the functional mapping relationship between sales quantity, sales price, and sales revenue. Neural networks have good correlation ability and should have better predictive ability for future sales [20]. To confirm this, we will use a trained neural network to predict the number of switch sales from 2017 to 2020.  Table 2 lists its specific prediction error values, and it is found that the average relative error of the neural network is only 0.9%. This can show that establishing a neural network sales forecast model is a feasible solution, and the prediction accuracy of this solution is quite high.

It can be seen from Table 2 that, compared with the linear regression method, the neural network method has higher accuracy and better prediction ability, and the accuracy of data prediction is also higher. It can be seen that the neural network method is better than the linear regression method in the sales test.

The article "Sales Forecast of Marketing Brand Based on BP Neural Network Model" was retracted in 2023. Reasons: signs of a paper mill; suspected computer-generated content; unreliable results or conclusions; concerns about the data.

The main products of the switch factory are plastic case circuit breakers (PCCB) and intelligent universal circuit breakers (IUCB). The monthly sales of these two products from 2015 to 2020 are shown in Tables 3 and 4.

As can be seen from Tables 3 and 4, whether it is ABC or MBCC, although the sales volume fluctuates, the overall trend is on the rise.

From the data shown in Tables 3 and 4, it can also be seen that the sales volume contains a long-term trend, random noise, and seasonal factors. This makes the accuracy of the data not high, so these data must be processed step by step before they can be used:

1. Data analysis and processing of ABC sales: It is necessary to understand the data that is generated by anomalous numerical points and noise. This part of the noise data is replaced by the average of the two-month sales numbers near the abnormal value point. The data considered outliers in these data can be replaced. These data points were averaged, and the processed data are shown in Table 5.
2. Data analysis and processing of MCCB sales. For MCCB, the analysis is the same as above. It removes various abnormal data in the original data that cannot reflect the changes in sales trends, and the data obtained after eliminating these points that are considered abnormal values, are shown in Table 6.

According to the model constructed above, the specific steps of using BP neural network to forecast the quarterly sales volume of switch factories in Shandong are as follows:

1. It selects the required sample data and builds a sample analysis model.
2. As of December 2020, this article counts sales for 24 quarters of 72 months. At the same time, we can see that when the total number of data points and the number of samples in each group are the same, if the learning rate of the network is too large (Ir = 0.8) or too small (Ir = 0.2), the number of network training rounds will increase. This is because a large learning rate makes the number of revisions too large, causing the weights to exceed the minimum value of some errors and regular jumps in the correction process, thus prolonging the number of exercises. However, a learning rate that is too small can produce very little modification, extending its learning time [21].
3. Data is classified into sample data and test data.
4. The samples are first classified, and the monthly sales volume before December 2019 is used as the training sample data, and the sales volume in the following year, 2020, is used as the test sample data for the neural network testing ability.
5. The sample data is preprocessed.
6. The data in the table is normalized according to the previous model and formula.
7. Sample training is conducted.
8. The data on the number of sales in each quarter is sequentially input to the network. It then uses the data of the next quarter as the data output by the network, that is, the target data. It arranges and combines the data in this way to form the sample data required for the neural network sales test.

The article "Sales Forecast of Marketing Brand Based on BP Neural Network Model" was retracted in 2023. Reasons: signs of a paper mill; suspected computer-generated content; unreliable results or conclusions; concerns about the data.

This results in a comparison of the predicted value, actual value, and errors for each month in 2020.

The sales volume of switch factory ABC and MBCC are forecast by neural network forecasting method and linear graphing method, respectively, to compare the errors of the two methods, specifically as shown in Figures 7–10.

It can be seen from Figures 7–10 that the neural network prediction is closer to the real data than the ordinary linear prediction, and its error is smaller. For comparison, a linear mapping method was used to predict the number of switches sold. First, the data is processed to eliminate unreasonable data and then analyzed and sorted, and finally a model of the number of switch sales is obtained. Neural network methods are used to create sales forecasting models. The neural network can approximate the value of the nonlinear function to any relatively accurate value. Therefore, it can also establish the functional mapping relationship between the sales quantity and other influencing factors, that is, sales price, product quality, etc. [22]. After the experiment, the prediction results show that it has higher approximation accuracy and better prediction ability than the conventional method (linear mapping method), and the prediction accuracy is more than 30% higher than that of the conventional method. Both models are predicting the short term, and the error of the prediction results is still acceptable. However, because of the small amount of data, the segmentation method makes the data of each segment too small. In each segment, the amount of data required by the neural network prediction method is insufficient, and the prediction effect has certain deficiencies. Predictions like ABC and MBCC's predictions for near term points are better. All of them can be used to guide the production of enterprises and so on and have certain practical application. However, there are also a few points with relatively large forecast errors, which are far from the actual sales.

## 5. Discussion

Globalization is the general trend. With the fast pace of globalization, most of the enterprises in China will have to engage in fierce competition in the international market, and these include manufacturing, transportation, and agriculture. To occupy the market in this fierce competition, we must speed up technological innovation, improve the technical content of products, and win the hearts of customers with high-quality services. However, the occupation of the market is definitely not so simple and subjective, and it depends on scientific and effective prediction. There are many studies on sales forecasting at home and abroad, but it is quite difficult to make scientific forecasts on sales in a complex economic situation. In BP neural network, in each round of model training, the weights are random. This makes the BP neural network not repeatable, resulting in strong randomness of the final model. Therefore, to improve the stability of the BP neural network's sales forecast results, we can consider combining other algorithms with neural networks to build a predictor with high stability of the forecast results.

The article "Sales Forecast of Marketing Brand Based on BP Neural Network Model" was retracted in 2023. Reasons: signs of a paper mill; suspected computer-generated content; unreliable results or conclusions; concerns about the data.

Through the analysis of the above two prediction models, it can be seen that for the prediction of the model obtained with 23 points, the errors obtained are quite different. Among them, the error predicted by the linear mapping method is larger. Therefore, it can be said that this model can be used for a specific enterprise or period, and if this model is widely used, it is necessary to analyze the specific application environment to obtain a more suitable prediction model. A simple evaluation and measurement of prediction results are discussed above, but in reality the work goes beyond that. The ultimate goal of predicting the results is to provide a highly reliable decision basis for the decision makers of the enterprise, so that they can make relatively scientific and correct decisions. Therefore, the requirement of predicting the results is to be as accurate as possible.

## 6. Conclusions

Since the beginning of the 21st century, the attention of enterprises to brands and their importance has reached an unprecedented level. All major companies are doing their best to build a strong brand. In addition, brand mergers and acquisitions have become one of the means of many companies. For example, China Southern Airlines merged with Central China Airlines, and Sanjiu Group acquired Long March Pharmaceuticals. However, acquisitions are only the first step toward owning a better brand. In the follow-up development, how to maintain and enhance the value of this brand is a more critical issue. This is also a relatively thorny problem that many companies are currently facing. The development of social economy and the intensification of market competition require enterprises to have very accurate market decision-making ability if they want to attract the attention of customers. Occupying the market does not mean that subjective assumptions are guaranteed to be effective. We must carefully study the mechanism of multiple market factors and use scientific methods to make accurate market forecasts on this basis. Only in this way can we ensure the success of a corporate strategy implementation. Artificial neural network is the most important theoretical basis of this paper. Thus far, the research in the field of artificial neural networks has spanned a history of nearly 60 years. Today, neural networks have become a hot and rapidly growing field of research. BP neural network has strong learning and associative memory capabilities, high fault tolerance, and a very strong nonlinear mapping function. When it is applied to the sales forecasting of enterprises, the forecasting accuracy is high and the generalization ability is good. Due to time and cost reasons, there are still many deficiencies in the marketing brand sales forecast model based on BP neural network established in this paper. In the experimental model, only a few factors that may affect brand sales are considered, which may bias the research results of BP neural network. Errors occur, and in future research, a more comprehensive consideration of factors affecting sales volume is required.

The article "Sales Forecast of Marketing Brand Based on BP Neural Network Model" was retracted in 2023. Reasons: signs of a paper mill; suspected computer-generated content; unreliable results or conclusions; concerns about the data.

## Figures and Tables

**Figure 1:** Neuron model diagram.

**Figure 2:** Schematic diagram of network topology.

**Figure 3:** Schematic diagram of Hopfield network topology.

**Figure 4:** Signal flow diagram of BP algorithm.

**Figure 5:** Schematic diagram of the single-layer neuron network model structure.

**Figure 6:** Schematic diagram of the three-layer neuron network model structure.

**Figure 7:** Comparison of ABC's monthly actual value and neural network prediction value and linear mapping prediction values in 2006.

**Figure 8:** Comparison of MBCC's monthly actual value and neural network prediction value and linear mapping prediction value in 2006.

**Figure 9:** Comparison of ABC's 2006 monthly neural network prediction error and linear prediction error.

**Figure 10:** Comparison of MBCC's 2006 monthly neural network prediction error and linear prediction error.

**Table 1:** Sales statistics of switch factories in the past 20 years.

Years	Sales	Price index	Income index
2001	10.2	91.8	232.4
2002	17.8	91.8	251.7
2003	18.5	93.6	244.9
2004	28.5	93.8	263.9
2005	51.7	94.3	296.5
2006	132.8	95.8	319.3
2007	249.2	91.6	339.7
2008	539.4	89.8	356.1
2009	592.3	97.2	385.6
2010	684.1	85.5	424.1
2011	1003.8	85.4	481.8
2012	1667.6	86.5	546.8
2013	1459.4	87.1	588.9
2014	1924.5	89.9	649.1
2015	2505.1	105.9	772.4
2016	2766.5	122.2	801.1
2017	2684.5	116.3	839.5
2018	2691.3	111.1	904.2
2019	2867.8	106.2	1034.4
2020	3032.8	108.2	1190.6

The article "Sales Forecast of Marketing Brand Based on BP Neural Network Model" was retracted in 2023. Reasons: signs of a paper mill; suspected computer-generated content; unreliable results or conclusions; concerns about the data.

**Table 2:** Comparison of prediction results and errors of the two methods.

Year	Actual value	Regression analysis			Neural network method		
		Predictive value	Absolute error	Relative error	Predictive value	Absolute error	Relative error
2017	2684.7	2150.9	-533.8	−19.88%	2731.5	46.8	1.74%
2018	2691.4	2746.8	55.4	2.06%	2768.1	76.7	2.85%
2019	2867.8	4046.5	1178.7	41.10%	2860.1	−7.7	−0.27%
2020	3032.9	5499.6	2466.7	81.33%	3011.5	−21.4	−0.71%
Average value	2819.2	3610.95	791.75	26.15%	2842.8	23.6	0.90%

*Note.* Absolute error = predicted value − actual value; relative error = absolute error/actual value.

**Table 3:** ABC sales.

Years	Monthly sales											
	The first quarter			The second quarter			The third quarter			The fourth quarter		
	January	February	March	April	May	June	July	August	September	October	November	December
2015	1	2	1	4	3	7	11	8	5	2	4	3
2016	3	6	8	7	14	5	16	29	9	11	6	3
2017	5	7	23	15	42	108	54	59	37	46	30	29
2018	36	21	17	69	52	49	163	43	32	23	19	41
2019	53	35	35	34	53	158	75	54	68	52	123	45
2020	28	74	46	92	208	89	84	104	90	85	52	64

**Table 4:** MBCC sales.

Years	Monthly sales											
	The first quarter			The second quarter			The third quarter			The fourth quarter		
	January	February	March	April	May	June	July	August	September	October	November	December
2015	34	18	186	145	619	503	409	97	125	156	64	127
2016	135	315	325	613	1636	770	774	740	290	339	234	371
2017	233	711	582	596	1314	3407	1778	3777	1037	1335	1115	1384
2018	1028	649	783	1510	3805	1691	1623	1192	1542	3906	1290	1712
2019	643	689	1119	917	1357	1015	1417	1109	1512	967	1171	2894
2020	1395	1245	2475	2749	2301	2067	1989	1833	1658	2035	1850	1749

**Table 5:** Data after ABC denoising.

Years	Monthly sales											
	The first quarter			The second quarter			The third quarter			The fourth quarter		
	January	February	March	April	May	June	July	August	September	October	November	December
2015	1	2	1	4	3	7	11	8	5	2	4	3
2016	3	6	8	7	14	5	16	29	9	11	6	3
2017	5	7	23	15	42	48	54	59	37	46	30	29
2018	36	21	17	69	52	49	47	43	32	23	19	41
2019	53	35	35	34	53	64	75	54	68	52	49	45
2020	28	36	46	92	90	89	84	104	90	85	52	64

**Table 6:** Data after MBCC denoising.

Years	Monthly sales											
	The first quarter			The second quarter			The third quarter			The fourth quarter		
	January	February	March	April	May	June	July	August	September	October	November	December
2015	34	18	186	145	619	503	409	97	125	156	64	127
2016	135	315	325	613	691	770	774	740	290	339	234	371
2017	233	711	582	596	1314	1545	1778	1407	1037	1335	1115	1384
2018	1028	649	783	1510	1601	1691	1623	1192	1542	1416	1290	966
2019	643	689	1119	917	1357	1015	1417	1109	1512	967	1171	1283
2020	1395	1245	2475	2749	2301	2067	1989	1833	1658	2035	1850	1749

The article "Sales Forecast of Marketing Brand Based on BP Neural Network Model" was retracted in 2023. Reasons: signs of a paper mill; suspected computer-generated content; unreliable results or conclusions; concerns about the data.

## Data Availability

The data that support the findings of this study are available from the author upon reasonable request.
